# An Effective Approach for Human Activity Classification Using Feature Fusion and Machine Learning Methods

**DOI:** 10.1155/2022/7931729

**Published:** 2022-02-02

**Authors:** Muhammad Junaid Ibrahim, Jaweria Kainat, Hussain AlSalman, Syed Sajid Ullah, Suheer Al-Hadhrami, Saddam Hussain

**Affiliations:** ^1^Department of Computer Science, University of Wah, 47040, Pakistan; ^2^Department of Computer Science, COMSATS University Islamabad, Wah Cantt, Pakistan; ^3^Department of Computer Science, College of Computer and Information Sciences, King Saud University, Riyadh 11543, Saudi Arabia; ^4^Department of Information and Communication Technology, University of Agder (UiA), N-4898 Grimstad, Norway; ^5^Computer Engineering Department, Engineering College, Hadhramout University, Hadhramout, Yemen; ^6^School of Digital Science, Universiti Brunei Darussalam, Jalan Tungku Link, Gadong BE1410, Brunei Darussalam

## Abstract

Recent advances in image processing and machine learning methods have greatly enhanced the ability of object classification from images and videos in different applications. Classification of human activities is one of the emerging research areas in the field of computer vision. It can be used in several applications including medical informatics, surveillance, human computer interaction, and task monitoring. In the medical and healthcare field, the classification of patients' activities is important for providing the required information to doctors and physicians for medication reactions and diagnosis. Nowadays, some research approaches to recognize human activity from videos and images have been proposed using machine learning (ML) and soft computational algorithms. However, advanced computer vision methods are still considered promising development directions for developing human activity classification approach from a sequence of video frames. This paper proposes an effective automated approach using feature fusion and ML methods. It consists of five steps, which are the preprocessing, feature extraction, feature selection, feature fusion, and classification steps. Two available public benchmark datasets are utilized to train, validate, and test ML classifiers of the developed approach. The experimental results of this research work show that the accuracies achieved are 99.5% and 99.9% on the first and second datasets, respectively. Compared with many existing related approaches, the proposed approach attained high performance results in terms of sensitivity, accuracy, precision, and specificity evaluation metric.

## 1. Introduction

In recent years, the e-vision community has focused largely on recognizing human activities. This is mainly because of a large number of industrial applications including human-computer interaction [1], antiterrorist applications [2], traffic surveillance [3], automotive safety [4], pedestrian detection [5], video surveillance [6], real-time tracking [7], rescue missions [8], and human-robot interaction [9]. This research work focuses on efficient recognition of human activity from recorded videos. Design of an efficient and optimal cost algorithm to detect a person from a video or an image is a challenging task. It is challenging in terms of variations of appearance, color, and movements [10]. Few other detection issues are also noticed like light and background variations [11]. Recently, numerous approaches have been proposed to detect a human from a video or an image. These approaches focused on the distinct use of classifiers, segmentation techniques, and feature extraction methods. Segmentation methods for human detection mainly contain foreground detection [12] and template matching [13]. Existing approaches do not yield optimal results with several humans in an image or a scene. Furthermore, there are many techniques used to detect humans like the Histogram of Gradients (HOG) [14], Haar-like features [15], adaptive contour features (ACF) [16], Hybrid Wind Farm (HWF) [17], Image Source Method (ISM) [18], edge detection [19], and movement characteristics [20]. These extraction methods do not clearly show the mark when people are unclear or have significant fluctuations in their positions. However, selections of relevant characteristics significantly improve human activity recognition. This research implemented a hybrid approach to overcome accuracy challenge of human activity identification. This is done by enhancing the quality of frames extracted from videos and later categorizing the regions on the basis of specified feature vectors. The approach proposed in this paper comprises of five major stages including (a) normalization, (b) feature extraction, (c) feature selection, (d) feature fusion, and (e) classification. Normalization is a preprocessing stage in which several techniques like background subtraction, noise removal, and object extraction are implemented. Three types of features are extracted which are HOG, Gabor, and chromatic features. Principal Component Analysis (PCA) is separately implemented on three feature vectors to get optimal features. Later, the serial feature fusion is incorporated on the selected features. Lastly, five versatile classifiers are applied to evaluate better accuracy.

### 1.1. Major Contributions

Inefficient and lengthy preprocessing procedures decline the optimality of any algorithm. This work focuses on the efficient and accurate use of preprocessing and feature extraction steps. Thus, main contributions in this work include the following:

- Morphological operations are applied after background subtraction to get the exact region of interest
- Separate principal component-based scoring for feature subset selection
- Optimal results are obtained by the application of multiple classification techniques

The chronological order of this manuscript is as follows: Section 1 provides domain introduction, Section 2 describes past work related to the recognition of the human activities, Section 3 describes the proposed method, and in Section 4, results are compared with other existing techniques.

## 2. Related Work

So much work has been done and is ongoing in human activity recognition. All of the approaches proposed lie under two main categories: (a) the traditional handcrafted feature extraction methods [21] and (b) the automatic features (deep learning) [22] which employ automatic feature extraction methods. Some major existing works performed in human activity recognition are discussed as follows: An activity recognition system based on streaming data is presented by Yala et al. [23]. The proposed technique efficiently detects significant human activities. Nunes et al. [24] presented a framework for daily human action recognition. The proposed technique firstly extracts various features. Later, every human activity frame is encircled by two consecutive automatically recognized key positions, in which maximum static and dynamic characteristics are extracted. Kantorov and Laptev [25] discovered feature encoding by Fisher vectors and determined accurate action recognition utilizing linear classifiers. Liu et al. [26] presented a framework in which multiple features are fused to make action recognition better. The proposed approach captures the silhouette deformation of the performer after considering activities as 3D objects. Azary and Savakis [27] use sporadic demonstrations of spatial and temporal aggregate movements with abnormal size and location characteristics. Oreifej and Liu [28] defined the depth order incorporating histogram that records the physical dispersion of the surface in the 4 dimensions including spatial, coordinates, depth, and time. Conde et al. [29] introduced a human crawling technique to watch videos that work in a dynamic environment. This approach used the combined function of HOG and Gabor [30].

In deep learning features, Wang et al. [31] proposed an algorithm which is useful to mine deep features from small video fragments. Additionally, depiction features of neighboring nodes of the secreted layer were considered according to similar activation states. Zhang et al. [32] introduced a less complex descriptor called 3D histogram texture in order to mine unique features from a given set of depth maps. On 3 orthogonal Cartesian planes, a three-dimensional histogram is formed. In [33], Lan et al. proposed an approach to influence operational methods from data-independent and data-driven methods to make action recognition systems better. Sargano et al. [34] proposed a new technique for recognizing human activity on the basis of the pretrained structure of the deep Convolutional Neural Network (CNN) for extraction and depiction of features in which the support vector machine (SVM) and *K*-Nearest Neighbor (KNN) are fused to recognize activity. In [35], the authors offered a small radial feature based on imaginary contour points and adapted to reactive real-time processing. Imaging-based features are useful for RGB-D images because of the shape, which is easily viewed as a bit mask based on the depth data provided by Microsoft Connect. Another common feature is presented by Tran and Sorokin [36]. It combines visual flow and silhouette into a single vector of attributes. With radial graphs, the silhouette and optical flow are encoded in *X*, *Y* dimensions and linked to a frame of fifteen adjacent frames. Lv and Nevatia [37] suggested a graph of the polynomial calculated by the selection of modified cell beams based on the logarithmic scale. Different kinds of human action include the abnormal activities by using the wireless connection. Support vector machine and the kernel nonlinear regression are used for reduction of the false positive rate. This can be done in the unsupervised learning. The proposed system performs the great function by using the real data [38]. Several techniques are used for finding the human activity in the videos. The authors worked on the feature correlation and frame differencing [39].

## 3. Proposed Methodology

In the proposed algorithm, a novel technique for human activity recognition is proposed. The proposed approach comprises of five basic steps, namely, these approaches are (a) detecting moving objects from the video sequence; (b) extracting the HOG, Gabor, and color features of the moving object; (c) selecting the best characteristics; (d) fusing the selected features serially; and (e) classifying the moving object.  Figure 1 shows the complete flow of the proposed technique.

### 3.1. Preprocessing

In the preprocessing stage, region-wise sliding window is implemented by considering variation in each consecutive frame. The needless regions including the background are ignored. A binary image is achieved after background subtraction on which the noise removal technique is applied. The binary image is transformed to RGB color space and later RGB is converted into Hue Saturation Intensity (HSI). In the next phase, a person is detected by drawing a bounding box around the person. The aim of preprocessing is to enhance the quality of video-extracted frames. The input image or frame extracted from a video is in RGB format. Preprocessing is applied to improve the foreground features for further processing. The steps of preprocessing are described below.

#### 3.1.1. Background Subtraction

Background subtraction is the first step in which RGB frames are extracted from the background and foreground videos for frame-by-frame processing. This is done because every processed frame gives us diverse results. With the presence of variations in every processed frame, the authenticity of the proposed algorithm is judged in a better way. In some cases, moving background or the presence of multiple objects is challenging to handle. The background frames are subtracted from the frames having a person doing a particular activity. Before taking the difference, both images are transformed from RGB color to HSI color. After that, the background image is subtracted from the actual image after converting from RGB to HSI. The conversion equation from RGB space and HIS space is given as [40]

(1) $$\begin{array}{c} I=\sqrt{3}\left(R+G+B\right), \end{array}$$

(2) $$\begin{array}{c} \theta =\arccos\frac{\left(1/2\right)\left[\left(R-G\right)+\left(R-B\right)\right]}{\sqrt{{\left(R-G\right)}^{2}+\left(R-B\right)\left(G-B\right.}}, \end{array}$$

(3) $$\begin{array}{c} H=\left\{\theta \;G\geq B\;2x-\theta \;G\leq B\right\}, \end{array}$$

(4) $$\begin{array}{c} S=1-\frac{3\;\min\;\left(R,G,B\right)}{R+G+B}, \end{array}$$

where *I*, *S*, and *H* are intensity, saturation, and hue, respectively. After this step, the binary image is produced. Some samples of the resulted images of this step can be seen in Figure 2(b).

#### 3.1.2. Morphological Operation

Images yielded after general background subtraction steps are noisy as shown in Figure 2(b). Morphological operation is applied to minimize the noise present in the image because the noisy image is not used for further processing. For this purpose, the preprocessing steps can be performed. The operation is known as opening by reestablishment of erosion, and it conserves the underlying shape of the object [41]. Regions having the least number of pixels are removed. The aim of this step is to detect the person in the image easily. After applying the opening morphological operation using the structuring element of 12-pixel-wide circular, the resulting images are much enhanced, and an individual is easily detected from the frame. The outcome of the enhanced image is shown in Figure 2(c). Hence, it is obvious that the opening morphological operation is the necessary step before object detection in the preprocessing stage.

#### 3.1.3. Image Cropping

Pixels from the white region in an image are counted to identify an object. The area which has more than 300 pixels is considered as the required object or human. All the white regions having less than 300 pixels are eliminated which are not required. When the object is detected, the bounding box is drawn around the person and the unnecessary part of the image is removed. The purpose of drawing the bounding box is to get the required part of the image by neglecting the unnecessary part as shown in Figure 2(d).

### 3.2. Feature Extraction

In the second stage of the proposed algorithm, three different types of extractors including HOG, Gabor, and cooccurrence matrices and chromatic features are employed to get the features of each frame. HOG, Gabor, and cooccurrence matrices and chromatic feature vectors are formed with 1 × 3780, 1 × 60, and 1 × 9 standard dimensions, respectively. Each feature is described as follows.

#### 3.2.1. HOG Features

In HOG feature extraction [14], the image is separated into small segments for individual processing. These segments are joined later. To achieve *G*_*x*_ and *G*_*y*_ directions, the Sobel kernel function is used on processed images. Mathematically, the process is depicted in the following equations.

(5) $$\begin{array}{c} F_{{\mathrm{seg}}_{\left|G\left(i,j\right)\right|}}=\sqrt{G_{x}{\left(i,j\right)}^{2}+G_{y}{\left(i,j\right)}^{2}}, \end{array}$$

(6) $$\begin{array}{c} F_{{\mathrm{seg}}_{\emptyset_{G}}}\left(i,j\right)=\tan-1\left(\frac{G_{y}\left(i,j\right)}{G_{x}\;\left(i,j\right)}\right), \end{array}$$

where ∣*G*∣ represents magnitude, ∅_*G*_ donates the angle of gradient, and *i* and *j* represent rows and columns simultaneously. The angle allocates the cell votes to bins based on the gradient. Later, the standardized vector is being achieved by using every block of the histogram. On the segmented image, the HOG feature descriptor is being implemented with 8 bin cells which are represented in the following equation.

(7) $$\begin{array}{c} F_{{{segV}^{N}}_{i}}=\frac{V_{i}}{\sqrt{\left({V_{2}}^{2}+{∊}^{2}\right)}}, \end{array}$$

where “∊” is a minor constant which does not divide by zero and *V* indicates the vector which is not normalized by containing all histograms in a block. When all of these vectors are combined in a single block, the HOG feature vector is achieved. Furthermore, mean variance and range through each feature are measured. Graphical representation of HOG features is shown in Figure 3.

#### 3.2.2. Gabor Features

In the spatial area, modified 2D-Gabor filter [42] is utilized using the “Gaussian Kernel” feature by a complex sinusoidal wave as shown in the following equation.

(8) $$\begin{array}{c} F_{\mathrm{seg}}=\frac{{fs}^{2}}{\pi Y\overset{\prime }{\eta }}\exp\left(-\frac{p^{\prime }+Y^{2}q^{\prime }}{2\sigma^{2}}\right)\exp\left(2\pi fsx^{\prime }+\emptyset \right). \end{array}$$

Here *fs* shows sinusoidal frequency, *θ* represents band similarity direction of an activity described by Gabor, ∅ indicates the phase offset, *σ* indicates the Standard Deviation (SD) of the Gaussian wrapper, and *Y* shows the characteristics regarding space proportion in which the elliptic support of the function described by Gabor is designated; *p*′ and *q*′ are described in the following equations.

(9) $$\begin{array}{c} x^{\prime }=x\text{coscos }\theta +y\text{sinsin }\theta , \end{array}$$

(10) $$\begin{array}{c} y^{\prime }=x\text{sinsin }\theta +y\text{coscos }\theta . \end{array}$$

Gabor feature [43] is implemented in six directions and five scales. Gabor feature measurement is chosen as 1 × 30. The variance and mean through the Gabor feature are measured. Graphical representation of HOG features is described in Figure 4.

#### 3.2.3. Cooccurrence Matrices and Chromatic Features

Grey tone spatial dependence is linked with cooccurrence technique. This approach works with the approximation. The function of the second-order density probability *h* (*i*, *j* | *d*, *θ*) is approximated. Each combined density function of the second order is calculated by measuring all pairs of pixels which are separated by distance *d* having gray levels *i* and *j* in the direction of the angle. The angular displacement *θ* is generally understood in the following interval: *θ* = {0, *π*/4, *π*/2, 3*π*/4}. The correlation table records a considerable amount of textual information. For a rough texture, these matrices usually have high values near the main diameter, while the costs are split into a soft texture. The cooccurrence matrices are summarized from the different directions to obtain a rotational invariant characteristic. This technique has become a reference point because of its intensive use [44], while other researchers relied on a smaller number of functions, such as entropy (*H*), correlation (COR), energy (*E*), and local homogeneity (LH).

(11) $$\begin{array}{c} E=\underset{i}{\sum }\underset{j}{\sum }{\left[h\left(i,j\;|\;d,\theta \right)\right]}^{2}, \end{array}$$

(12) $$\begin{array}{c} H=-\underset{i}{\sum }\underset{j}{\sum }\left[h\left(d,\theta \right)\;\log\;h\left(d,\theta \right)\right], \end{array}$$

(13) $$\begin{array}{c} I=\underset{i}{\sum }\underset{j}{\sum }\left[{\left(i-j\right)}^{2}\;h\left(d,\theta \right.\right], \end{array}$$

(14) $$\begin{array}{c} \text{LH}=\underset{i}{\sum }\underset{j}{\sum }\frac{\left(i,j\;|\;d,\theta \right)}{1+{\left(i+j\right)}^{2}}, \end{array}$$

(15) $$\begin{array}{c} \text{COR}=\underset{i}{\sum }\underset{j}{\sum }\frac{\left(i-\mu_{x}\right)\left(j-\mu_{y}\right)\;h\left(i,j\;|\;d,\theta \right)}{\sigma_{x}\sigma_{y}}, \end{array}$$

where *μ*_*x*_ is the horizontal mean, *σ*_*x*_ is the variance, and both *μ*_*y*_ and *σ*_*y*_ are the vertical statistics.

This technique records second-degree grayscale statistics related to human perception and texture discrimination which are used with various disadvantages [45]. The disadvantage of the given technique is that it does not explain the aspects of the shape and type of texture. In addition, this technique involves choosing an appropriate level of quantification. Text information may be lost due to the reduced number of antenna sizes at the quantization level. And a relatively large number of compartments can lead to irrelevant text features.

### 3.3. Feature Selection

The sensitivity of various machine defect features differs meaningfully in dissimilar working circumstances. It becomes vital to develop an organize feature selection structure. This provides the basis for organization of descriptive structures [46]. In the proposed technique, PCA is used for feature selection to select the prominent features separately from the results of HOG, Gabor, and cooccurrence matrices and chromatic feature vectors.

Generally, the PCA method converts from *d*-dimensional space of *n* vectors to another space of *d*′-dimensions having *n* vectors (*x*_1_′, *x*_2_′, ⋯, *x*_*i*_′, ⋯, *x*_*n*_′) as given by the following equation [47].

(16) $$\begin{array}{c} x_{r}^{\prime }=\overset{d^{\prime }}{\underset{n=1}{\sum }}a_{n,r}e_{n},\;d^{\prime }\leq d, \end{array}$$

where *e*_*n*_ shows the eigenvectors relating with *d*′-dimensional space and largest eigenvalues of the disseminated matrix *S*. On the other hand, *a*_*n*,*r*_ are forecasts of the vectors *xr* on the eigenvectors. These are the main constituents of true datasets. The *d* and  *d*′ are both positive integers such that *d*′ cannot be greater than *d* in any of the cases. *d* × *d* matrix *S* represents the original dataset (*x*_1_, *x*_2_, ⋯, *x*_*i*_, ⋯, *x*_*n*_) which is defined as

(17) $$\begin{array}{c} S=E\left[x_{i}x_{i}^{T}\right],\;\text{for }i=1\text{ to }n, \end{array}$$

where *E*[*x*_*i*_*x*_*i*_^*T*^] is the “statistical expectancy operator” implemented on the external multiplicative product of *x*_*i*_ and  *x*_*i*_^*T*^. The depiction illustrated in Equation (26) decreases the occurrence of error between the converted vectors and the original. If the variance of principal components such as  (*a*_*n*,*r*_)  is considered, the problem is simplified.

### 3.4. Feature Fusion

The purpose of feature fusion makes the action recognition algorithm efficient. This also enhances the action classification rate of human in complicated scenarios. In this method, feature fusion produces considerably improved results not only in the dark background but also in the high brightness environment as compared to original Gabor and HOG features. Hand-crafted features are combined with the deep learning models. The model is named as the posteriori algorithm [48].

For fusing the features, a unique method is deployed which depends on the vector dimension size. The size of these feature vectors are 1 × 60, 1 × 3780, and 1 × 9 in HOG, Gabor, and cooccurrence matrices and chromatic features, respectively. For feature fusion, let *C*_1_, *C*_2_, *C*_3_, ⋯, *C*_*n*_ be the human activity classes, which need to be classified. Let Δ = {∅v∅∈RN} indicate the number of training samples. {*Ύ*_HOG_, *Ύ*_Gab_, *Ύ*_Chrom_} ∈ *R*^*N*_*HOG*+*Gab*+*Chrom*_^ are the three feature vectors extracted. The size is defined as

(18) $$\begin{array}{c} {\text{FV}}_{1}=\left\{j_{1},\cdots j_{k}\right\},{\text{FV}}_{2}=\left\{y_{1},\cdots y_{k}\right\},{\text{FV}}_{3}=\left\{d_{1},\cdots d_{k}\right\}, \end{array}$$

where FV_1_, FV_2_, and FV_3_ indicate the size of HOG, Gabor, and cooccurrence matrices and chromatic features, respectively. The sizes of the feature vectors are characterized through set *k*, where *k* ∈ {60, 3780, 9}. As discussed earlier, the sizes of extracted feature sets are (′*ϒ*_HOG_⟶1 × 3780,  ′*ϒ*Gab⟶1 × 60,  ′*ϒ*Chrom⟶1 × 9). The final extracted vector is indicated as

(19) $$\begin{array}{c} F\left(\emptyset \right)=\overset{{\text{FV}}_{1}}{\underset{j}{\sum }}{Ύ}_{\text{HOG}}+\overset{{\text{FV}}_{2}}{\underset{t}{\sum }}{Ύ}_{\text{Gab}}+\overset{{\text{FV}}_{3}}{\underset{d}{\sum }}{Ύ}_{\text{Chrom}}, \end{array}$$

(20) $$\begin{array}{c} F\left(\emptyset \right)=\left\{\left(1\times 3780\right)+\left(1\times 60\right)+\left(1\times 9\right)\right\}, \end{array}$$

(21) $$\begin{array}{c} \text{Final }\left(\emptyset \right)=\left\{1\times 3849\right\}. \end{array}$$

### 3.5. Classification

Five different classifiers including linear-SVM, cubic-SVM, complex tree, fine-KNN, and subspace-KNN are used for result comparisons.  Figure 5 depicts the detailed view of feature selection, fusion, and selection.

The accuracy achieved by subspace-KNN is highest among all the classifiers on the KTH dataset, while cubic-SVM has achieved higher accuracy than other classifiers on the Weizmann dataset. The random subspace approach depends on a stochastic procedure which selects the components of the particular feature vector randomly to construct every classifier. In the KNN classifier, when a testing sample is compared to the original, only the chosen features will get the nonzero contributions [49]. On the other hand, State Vector Machines construct models which are complicated and contain radial basis function (RBF), polynomial classifiers, and large neural nets. It is easy to examine mathematically; it resembles a linear method in a multidimensional feature space nonlinearly associated with the input space [50].

## 4. Results and Analysis of Experiment

The experimental setups, datasets, and results based on the performance measures are discussed in this section.

### 4.1. Experimental Setup

The time elapsed during activity classification depends on resources such as memory, Central Processing Unit (CPU) speed, power supplies, disk storage, and cooling systems. This can precisely describe a linear relationship between elapsed time and CPU usage. The tested system (DELL Latitude E5520) to run the proposed algorithm consists of a Microsoft Windows 10 Pro environment with Intel Core-i5 2540M @ 2.60 GHz processor. The system RAM is 4.00 GB with a 64-bit operating system and an x64 processor. All the results presented in this section are the results obtained in this system.

### 4.2. Datasets

To validate the results, two different types of datasets are used in this research. This includes KTH and Weizmann datasets. Both of the datasets are described briefly hereunder.

#### 4.2.1. Weizmann Dataset

The Weizmann dataset [51] contains 2513 human activity images. It covers five types of human behavior performed by nine different actors. To verify the proposed algorithm, a 50 : 50 method is run. This means that half of the images are used for training the classifier and the remaining half are used to test the performance of the algorithm. After the selection and fusion of features, classification techniques are applied to evaluate the results.  Figure 6 shows some images as a sample from the Weizmann dataset.

#### 4.2.2. KTH Datasets

KTH datasets consists of 1628 images of six different types of human activities. Images with different variations are chosen for the authentication of the proposed method. Half of the images are used in the training of the classifier while the remaining 50% are used for the purpose of testing.  Figure 7 shows some of the images from the Weizmann datasets. These datasets include boxing, clapping, hand waving, running, and walking.

### 4.3. Performance Measures

Performance of the proposed algorithm is assessed on the basis of performance measures such as specificity (SPE), area under the curve (AUC), precision (PRE), sensitivity (SEN), and accuracy (ACU). Mathematically, it is represented by the following equations.

(22) $$\begin{array}{c} \text{PRE}=\frac{\text{TP}}{\text{TP}+\text{FP}}, \end{array}$$

(23) $$\begin{array}{c} \text{SEN}=\frac{\text{TP}}{\text{TP}+\text{FN}}, \end{array}$$

(24) $$\begin{array}{c} \text{SPE}=\frac{\text{TN}}{\text{TN}+\text{FP}}, \end{array}$$

(25) $$\begin{array}{c} \text{ACU}=\frac{\text{TP}+\text{TN }}{\text{FP}+\text{TP}+\text{FN}+\text{TN}}, \end{array}$$

(26) $$\begin{array}{c} \text{AUC}=\int_{\infty }^{-\infty }\frac{\text{TPR}\left(T\right)\text{FPR}}{\left(T\right)dT}. \end{array}$$

In the above equations, FP represents false positive, TN represents true negative, TP represents true positive, and FN represents false negative.

All of the performance measures mentioned in Equation (20) to (25) are calculated from confusion matrices. These matrices have the finest results of the Weizmann and KTH datasets.

### 4.4. Experiments

For quantitative outcomes, six different experiments are implemented using a separate number of features. The comprehensive description of all experiments with a numeral classes, numeral folds, and features can be seen in Table 1. The comprehensive analyses of experiments performed on 316 bend, 624 hand waving, 457 jumping, 405 run, and 711 walk images are described in the upcoming sections.

#### 4.4.1. Experiment 1: Shape Features—100, Texture Features—60, and Color Features—9

In experiment 1, a total of 2513 and 1628 images are collected from the Weizmann and KTH datasets, respectively. The Weizmann dataset consists of 5 categories of manual bending, jumping, running, and walking images, while the KTH dataset includes 6 classes which are clapping, boxing, running, hand waving, and walking. To get the experimental results, 50% of images are used for the purpose of training and the remaining 50% of them are used for testing. For assessment of the results, the “5-fold” validation is used. For experiment 1, the maximum classification rate is 99.3% for the Weizmann dataset obtained with cubic-SVM. The linear-SVM and subspace-KNN obtained 99.8% accuracy simultaneously on the KTH dataset as shown in Table 2. Cubic-SVM obtained a better sensitivity rate of 98.84, specificity of 99.81 and accuracy of 98.98 as compared to other classification methods using the Weizmann dataset. On the other hand, linear-SVM and subspace-KNN obtained a sensitivity rate of 99.86, specificity of 99.96, and precision of 98.74 which is better in comparison with other classification methods using the KTH dataset.

#### 4.4.2. Experiment 2: Shape Features—300, Texture Features—60, and Color Features—9

In experiment 2, 2513 and 1628 images are taken from the Weizmann and KTH datasets, respectively. The Weizmann dataset includes five categories. These five categories are bending, handshaking, jumping, running, and walking, while the KTH dataset includes 6 classes which are boxing, clapping, handshake, jogging, running, and walking. For experimental results, half of the images from each dataset are used for training and the remaining half are used for the purpose of testing. For assessment of the results, “10-fold” validation is used. The 10-fold validation is known as the evaluation method. For experiment 2, the maximum classification frequency is 99.5% for the Weizmann dataset on cubic-SVM, while for the KTH dataset, 99.9% is achieved in the subspace-KNN, as shown in Table 3. The cubic-SVM applied to the Weizmann dataset is better in terms of sensitivity of 99.34, specificity of 99.89, and precision of 99.5 than other approaches, whereas the KNN subdomain applied to the KTH dataset is better in terms of sensitivity of 99.97, specification of 99.99, and accuracy of 99.95 than the other classification approaches.

The experiment 2 produces the best results among all the five experiments implemented during this research process. The proposed algorithm produced the best results on the conditions provided in the experiment 2. The best results calculated on the basis of performance measures of the KTH and Weizmann datasets using confusion matrices are shown in Tables 4 and 5, respectively. The KTH datasets give 99.9% accuracy using the subspace-KNN classifier and the Weizmann dataset produced 99.5% accuracy using cubic-SVM which is best among all other classifiers.

#### 4.4.3. Experiment 3: Shape Features—500, Texture Features—60, and Color Features—9

In experiment 3, a total of 2513 images of the Weizmann dataset and 1628 images of the KTH dataset are collected. Five classes from the Weizmann dataset are selected which includes bending, hand waving, jumping, running, and walking. Six classes from the KTH dataset including clapping, boxing, running, hand waving, walking, and hand waiving are selected.

For experimental results, half of images from both datasets are selected for training purposes and the remaining half are used for testing. For assessment of the results, “8-fold” validation is used. Maximum classification frequency attained on cubic-SVM is 98.7% for the Weizmann datasets. For the KTH datasets, 99.9% accuracy is attained on subspace-KNN as given in Table 6. The cubic-SVM implemented for the Weizmann datasets is better in terms of sensitivity of 97.86, specificity of 99.67, and precision of 98.54 as compared to other approaches. On the other hand, the subspace-KNN implemented for the “KTH” datasets is better in terms of sensitivity of 99.97, specificity of 99.99, and precision of 99.95 as compared to other approaches.

#### 4.4.4. Experiment 4: Shape Features—800, Texture Features—59, and Color Features—9

In experiment 4, total of 2513 images of Weizmann datasets and 1628 images of KTH datasets are collected. The Weizmann datasets are comprised of 5 classes including bending, hand waving, jumping, running, and walking images. The KTH datasets are comprised of 6 classes including clapping, boxing, running, hand waving, walking, and hand waiving. For experimental results, half of images from both the datasets are selected for training and the other half of them are used for testing. For assessment of the results, “5-fold” validation is used. Maximum classification frequency of 95.9% for the Weizmann datasets is attained on linear-SVM while 99.9% for the KTH dataset on subspace-KNN as given in Table 7. The linear-SVM implemented for the Weizmann dataset is better in terms of sensitivity of 93.38, specificity of 98.96, and precision of 96.09 from other approaches. On the other hand, the subspace-KNN implemented for the “KTH” dataset is better in terms of sensitivity of 99.97, specificity of 99.99, and precision of 99.45 from other approaches.

#### 4.4.5. Experiment 5: Shape Features—1100, Texture Features—55, and Color Features—9

In experiment 5, a total of 2513 images of the Weizmann dataset and 1628 images of the KTH dataset are collected. The Weizmann dataset comprising of 5 classes including bending, hand waving, jumping, running, and walking images is selected. The KTH dataset comprising of 6 classes including clapping, boxing, running, hand waving, and walking is selected. For experimental results, half of the images from both datasets is selected for training the algorithm and the remaining half is used for testing. For appraisal of the results, “7-fold” validation is used. Maximum classification frequency is 92.0% for the Weizmann datasets on subspace-KNN while 99.9% for the KTH dataset on subspace-KNN as given in Table 8. The class-wise AUCs are mentioned in Table 9. The subspace-KNN implemented for the Weizmann datasets is better in terms of sensitivity of 88.72, specificity of 97.96, precision of 90.81, and AUC. We can say that subspace-KNN gives the better results. On the other hand, the subspace-KNN implemented for “KTH” datasets is better in terms of sensitivity of 99.97, specificity of 99.99, and precision of 99.95. The results of experiment 5 are presented in Table 8.

## 5. Discussion

This section presents a detailed analysis of experimental outcomes through the proposed method on the basis of accuracy measures such as precision, sensitivity, specificity, and accuracy. The proposed algorithm consists of five main stages. These five main stages include the preprocessing which is performed first in which datasets are normalized to get better results. The accurate results will give more accuracy. In the second step, feature extraction is implemented using HOG, Gabor, and chromatic feature extractor. In the third step, feature selection is implemented separately based on PCA to get the best features. In the fourth step, features are fused, while in the final stage, results are taken through the classification learner. In preprocessing, background subtraction is done to detect the human from the image and the noise is removed using morphological operations. After removing the noise, a bounding box is drawn to around the person to ignore the unnecessary parts using cropping. In the next step, three kinds of features comprising shape, texture, and color are extracted from segmented images. Five classifiers containing linear-SVM, cubic-SVM, complex tree, fine-KNN, and subspace-KNN are used to test the proposed algorithm. Subspace-KNN and cubic-SVM have achieved higher accuracy than the other classification learners on the “Weizmann” and “KTH” datasets, respectively.

In the experimental results, six classes of KTH datasets and five classes of Weizmann datasets are used to get results. 99.90% and 99.5% accuracies for KTH datasets using subspace-KNN are achieved using subspace-KNN and cubic-SVM, respectively. Comparison of the previously implemented algorithms with the proposed algorithm is shown in Table 10. The table is explained in a better way. On the basis of the above discussion, it is clear that the combination of three feature extractors used in the proposed algorithm gives better accuracy as compared to the already implemented algorithms.

## 6. Conclusion

In this research, a technique is proposed for the “detection” and “classification” of several activities from videos and multimedia frames. The proposed algorithm consists of five pipeline processes which are preprocessing, feature extraction, feature selection, serial feature fusion, and classification. From all results shown above and in Discussion, it is obvious that by using the proposed technique, the detection of human activities is tackled. Five different experiments are executed to judge the authenticity of this algorithm. The results of all five experiments are discussed in detail in Results and Analysis of Experiment. The KTH and Weizmann datasets are selected to check the reliability of this algorithm. This method executed better on the KTH and Weizmann datasets. Moreover, it is determined that shape features are very important for the classification of chosen classes such as bending, jumping, running, walking, and hand waving. The texture and color features are very essential for the detection and classification of different usual activities performed by a human being. To enhance the system performance, feature selection and feature fusion seem to be quite significant as accuracy and sensitivity. In contrast to the existing techniques, the proposed technique has achieved higher accuracy which is 99.9% on KTH datasets and 99.5% on Weizmann datasets.

## Figures and Tables

**Figure 1:** Detailed description of proposed model based on the machine learning methods.

**Figure 2:** Preprocessing stages: (a) original images; (b) background subtraction images; (c) image enhancement; (d) object detection; (e) binary to RGB conversion; (f) image cropping.

**Figure 3:** Visualization of histogram of oriented gradient features: (a) original image; (b) HOG features.

**Figure 4:** Gabor feature visualization: (a) original image; (b) Gabor features.

**Figure 5:** Feature vector selection, fusion, and classification.

**Figure 6:** Sample images of Weizmann dataset.

**Figure 7:** Sample images of KTH dataset.

**Table 1:** Summary of experiments setting for Weizmann and KTH datasets.

Exp no.	No. of classes		Shape	Texture	Color	Folds
	KTH	Weizmann				
1	6	5	100	60	9	5
2	6	5	300	60	9	10
3	6	5	500	60	9	8
4	6	5	800	58	9	5
5	6	5	1100	55	9	7

**Table 2:** Classification results of experiment 1 with all possible values.

Weizmann					KTH			
Method	SEN (%)	SPE (%)	PRE (%)	ACU (%)	SEN (%)	SPE (%)	PRE (%)	ACU (%)
Linear-SVM	98.8	99.7	98.52	98.8	99.85	99.95	99.03	99.8
Cubic-SVM	98.84	99.81	98.98	99.3	99.8	99.94	99.09	99.7
Complex tree	85.92	97.33	86.06	89.0	98.26	99.67	97.77	98.4
Fine-KNN	98.99	99.78	99.23	99.0	99.77	99.91	99.75	99.6
Subspace-KNN	90.3	98.30	91.7	93.3	99.86	99.96	99.74	99.8

**Table 3:** Classification results of experiment 2 along with the sensitivity and other measures.

Weizmann					KTH			
Method	SEN (%)	SPE (%)	PRE (%)	ACU (%)	SEN (%)	SPE (%)	PRE (%)	ACU (%)
Linear-SVM	98.83	99.84	99.0	99.3	99.89	99.95	99.89	99.8
Cubic-SVM	99.34	99.89	99.5	99.5	98.81	99.94	98.60	99.7
Complex tree	85.40	97.15	85.0	88.3	98.32	99.67	97.37	98.5
Fine-KNN	87.26	97.21	95.4	91.1	99.42	99.84	99.38	99.2
Subspace-KNN	90.25	98.3	91.9	93.9	99.97	99.99	99.95	99.9

**Table 4:** Confusion matrix of KTH dataset of experiment 2 on subspace-KNN.

Classification classes	Total images	Clapping	Jogging	Hand waving	Running	Walking	Boxing
Clapping	312	312					
Jogging	191		191				
Hand waving	581	1		580			
Running	109				109		
Walking	27					27	
Boxing	408						408

**Table 5:** Confusion matrix of Weizmann dataset of experiment 2 on cubic-SVM.

Classification classes	Total images	Hand waving	Running	Jumping	Walking	Bending
Hand waving	624	624				
Running	206		201	2	3	
Jumping	421	1		420		1
Walking	271		2	2	267	
Bending	375					375

**Table 6:** Classification results of experiment 3 using the linear-SVM method and others.

Weizmann					KTH			
Method	SEN (%)	SPE (%)	PRE (%)	ACU (%)	SEN (%)	SPE (%)	PRE (%)	ACU (%)
Linear-SVM	97.90	99.69	98.39	98.7	100	99.72	98.70	98.7
Cubic-SVM	97.86	99.67	98.544	98.7	91.51	99.21	96.39	96.5
Complex tree	85.43	97.212	85.53	88.6	98.34	99.69	97.93	98.5
Fine-KNN	63.7	91.63	90.79	71.9	95.30	99.32	98.02	97.0
Subspace-KNN	89.99	98.18	92.11	93.0	99.97	99.99	99.95	99.9

**Table 7:** Classification results of experiment 4.

Weizmann					KTH			
Method	SEN (%)	SPE (%)	PRE (%)	ACU (%)	SEN (%)	SPE (%)	PRE (%)	ACU (%)
Linear-SVM	93.38	98.96	96.09	95.9	59.25	96.7	90.90	85.3
Cubic-SVM	91.56	98.5	95.63	94.5	57.56	96.45	74.49	84.3
Complex tree	80.56	97.18	85.57	88.5	97.74	99.63	97.51	98.2
Fine-KNN	46.29	87.54	88.81	58.2	70.14	96.30	90.90	84.0
Subspace-KNN	89.21	98.37	91.44	92.5	99.97	99.99	99.45	99.9

**Table 8:** Classification results of experiment 5.

Weizmann					KTH			
Method	SEN (%)	SPE (%)	PRE (%)	ACU (%)	SEN (%)	SPE (%)	PRE (%)	ACU (%)
Linear-SVM	80.0	96.68	90.0	87.5	50.83	95.49	57.16	80.2
Cubic-SVM	80.0	96.20	90.31	86.3	50.42	95.37	55.03	79.5
Complex tree	85.32	97.8	85.31	88.4	98.49	99.69	97.93	98.6
Fine-KNN	33.42	84.1	87.63	46.7	39.47	93.6	84.92	57.6
Subspace-KNN	88.72	97.96	90.81	92.0	99.97	99.99	99.95	99.9

**Table 9:** AUC results.

Method	Classes	Experiment 1		Experiment 2		Experiment 3		Experiment 4		Experiment 5	
		Weizmann	KTH	Weizmann	KTH	Weizmann	KTH	Weizmann	KTH	Weizmann	KTH
Linear-SVM	C1 C2 C3 C4 C5 C6	1.00 0.99 1.00 1.00 1.00	1.00 1.00 1.00 1.00 1.00 1.00	1.00 1.00 1.00 1.00 1.00	1.00 1.00 1.00 1.00 1.00 1.00	1.00 1.00 1.00 1.00 1.00	1.00 1.00 1.00 1.00 0.98 1.00	1.00 0.99 1.00 0.99 1.00	1.00 0.98 1.00 0.99 1.00 1.00	1.00 0.98 0.99 0.98 1.00	1.00 0.90 1.00 0.98 1.00 1.00
Cubic-SVM	C1 C2 C3 C4 C5 C6	1.00 1.00 1.00 1.00 1.00	1.00 1.00 1.00 1.00 1.00 1.00	1.00 1.00 1.00 1.00 1.00	1.00 1.00 1.00 1.00 1.00 1.00	1.00 1.00 1.00 1.00 1.00	1.00 1.00 1.00 1.00 0.99 1.00	1.00 0.99 1.00 0.99 1.00	1.00 0.98 1.00 0.99 0.99 1.00	1.00 0.98 0.99 0.98 1.00	1.00 0.90 1.00 0.98 1.00 0.99
Complex tree	C1 C2 C3 C4 C5 C6	0.98 0.87 0.94 0.90 0.97	1.00 0.98 1.00 0.99 0.98 1.00	0.99 0.89 0.93 0.88 0.95	1.00 0.96 1.00 0.98 0.96 1.00	0.98 0.85 0.94 0.90 0.97	1.00 0.98 1.00 0.99 0.98 1.00	0.98 0.88 0.94 0.88 0.96	0.99 0.99 0.99 0.99 1.00 1.00	0.98 0.87 0.94 0.87 0.96	0.99 0.99 0.99 0.96 1.00 1.00
Fine-KNN	C1 C2 C3 C4 C5 C6	1.00 0.99 0.99 0.99 1.00	0.98 1.00 0.98 0.81 1.00 0.98	0.93 0.87 0.91 0.92 1.00	0.97 1.00 0.99 0.69 1.00 0.96	0.79 0.63 0.71 0.76 0.99	0.98 0.99 0.98 0.64 1.00 0.94	0.69 0.51 0.65 0.61 0.89	0.95 0.88 0.91 0.61 0.76 0.91	0.60 0.50 0.62 0.51 0.71	0.75 0.54 0.76 0.50 0.54 0.81
Subspace-KNN	C1 C2 C3 C4 C5 C6	1.00 0.98 1.00 0.99 1.00	1.00 1.00 1.00 1.00 1.00 1.00	1.00 0.98 0.99 0.99 1.00	1.00 1.00 1.00 1.00 1.00 1.00	1.00 0.98 1.00 0.99 1.00	1.00 1.00 1.00 1.00 1.00 1.00	1.00 0.98 0.99 0.99 1.00	1.00 1.00 1.00 1.00 1.00 1.00	1.00 0.98 1.00 0.99 1.00	1.00 1.00 1.00 1.00 1.00 1.00

**Table 10:** Comparison of action recognition results.

Reference	Year	Recognition (%)
*Weizmann dataset*		
[52]	2013	95.45
[53]	2014	95.56
[54]	2015	95.10
[55]	2016	88.10
[7]	2017	95.80
[56]	2019	99.0
[57]	2020	96.0
Proposed	2018	99.5
*KTH dataset*		
[58]	2014	95.0
[59]	2015	95.21
[60]	2015	96.50
[61]	2016	97.10
[62]	2017	94.92
[7]	2017	99.30
[63]	2020	94.83
[64]	2019	91.67
Proposed	2018	99.90

## Data Availability

The data used to support the findings of this study are available from the corresponding author upon request.
